# Influence of Standardized Nursing Intervention Combined with Mindfulness Stress Reduction Training on the Curative Effect, Negative Emotion, and Quality of Life in Patients with Chronic Gastritis and Gastric Ulcer

This article has been retracted.

**DOI:** 10.1155/2021/2131405

**Published:** 2021-10-14

**Authors:** Hongmei Xiao, Zhibin Zhao, Cuijuan Zhang, Jimin Wang

**Affiliations:** ^1^Department of Gastroenterology, Taizhou People's Hospital, Taizhou, Jiangsu 225300, China; ^2^Department of Traditional Chinese Medicine, Xiangyang Central Hospital, Affiliated Hospital of Hubei University of Arts and Science, 441021 Xiangyang, Hubei, China

## Abstract

**Objective:**

To explore the curative effect of standardized nursing intervention combined with mindfulness stress reduction training in patients with chronic gastritis and gastric ulcer and its influence on negative emotion and quality of life.

**Methods:**

Total of 146 patients with chronic gastritis and gastric ulcer admitted to our hospital from August 2018 to February 2020 were collected and divided into the control group (*n* = 73) and study group (*n* = 73) according to patients' wishes and the random number method. The control group received traditional nursing measures. The study group received standardized nursing intervention combined with mindfulness stress reduction training. The general data, nursing efficiency, negative emotions, self-efficacy, quality of life, and nursing satisfaction of the two groups were recorded.

**Results:**

The nursing effective rate of the study group (91.78%) was higher than the control group (79.45%) (*P* < 0.05). After intervention, the self-rating anxiety scale score and self-rating depressive scale score of the study group were lower than the control group (*P* < 0.05). After intervention, the general self-efficacy scale score and the generic quality of life inventory-74 scores of the study group were higher than the control group (*P* < 0.05). The nursing satisfaction rate of the study group (89.04%) was higher than the control group (75.34%) (*P* < 0.05).

**Conclusion:**

Standardized nursing intervention combined with mindfulness stress reduction training has a good curative effect in patients with chronic gastritis and gastric ulcer, which is beneficial to reduce negative emotions, increase self-efficacy, improve quality of life, and improve nursing satisfaction.

## 1. Introduction 

Chronic gastritis and gastric ulcer have become common digestive tract diseases in the clinic, which are mostly caused by *Helicobacter pylori* infection, excessive mental stress, irregular diet, poor living habits, food stimulation, smoking, and alcoholism [1]. Chronic gastritis refers to chronic inflammatory lesions of gastric mucosa caused by various factors. Chronic gastritis can be diagnosed by gastroscopy, and its incidence ranks first among various stomach diseases [2]. Gastric ulcer is an ulcer caused by the damage of the mucosal muscle layer caused by gastric acid digestion of gastrointestinal mucosa. In severe cases, it may cause serious consequences such as gastric bleeding, pyloric obstruction, and canceration [3]. The most common clinical manifestations of chronic gastritis and gastric ulcer are stomach pain, abdominal distention, acid regurgitation, nausea, belching, loss of appetite, and other symptoms, and their frequent attacks bring great harm to the patients' daily life. At present, the incidence of chronic gastritis and gastric ulcer in men is higher than that in women, and the disease can occur at all ages. However, in recent years, the incidence age of gastrointestinal diseases tends to be younger. Because the etiology of chronic gastritis and gastric ulcer is complex, the onset is slow, the course of disease is prolonged, and the patients often suffer from different degrees of physiological discomfort, which easily leads to a variety of negative psychology, thus aggravating the degree of illness, reducing compliance, and affecting physical and mental health, which is not conducive to the treatment effect of patients [4]. Therefore, it is of great significance to take scientific and reasonable intervention measures for patients with chronic gastritis and gastric ulcer in time.

Standardized nursing belongs to a nursing method integrating nursing, psychology, medicine, and other disciplines. It is an intervention method that takes the patient as the core and gives comprehensively and meticulously care for every detail of the patient's physiology and psychology [5]. Standardized nursing has the characteristics of unity and flexibility, which can significantly improve patients' compliance behavior, improve clinical symptoms of diseases, enhance patients' body functions, and then promote patients' early recovery [6]. Mindfulness stress reduction training was born in 1979 and founded by Dr. Kabat-Zinn. Mindfulness stress reduction training, as a special psychological adjustment method, can assist general medical behavior to effectively improve people's psychological state and has been widely used in the clinic [7]. Mindfulness stress reduction training aims to teach patients to mobilize their physical and mental strength through meditation, breathing, body scanning, and other measures to increase the mindfulness feedback to their body and mind and to guide patients to devote themselves and accept themselves without criticism, so as to enhance cognitive ability, relieve disease pain, relieve inner pressure, and promote disease recovery [8].

According to literature search, there is no research report on the effect of standardized nursing intervention combined with mindfulness stress reduction training on patients with chronic gastritis and gastric ulcer at this stage. Our physicians have extensive nursing experience. Through standardized nursing intervention combined with mindfulness stress reduction training for 73 patients with chronic gastritis and gastric ulcer, we observed their negative emotions and quality of life, in order to provide a new choice for the application of clinical nursing programs.

## 2. Methods

### 2.1. Research Object

Total of 146 patients with chronic gastritis and gastric ulcer admitted to our hospital from August 2018 to February 2020 were collected and divided into the control group (*n* = 73) and study group (*n* = 73) according to patients' wishes and the random number method. Inclusion criteria: chronic gastritis and gastric ulcer diagnosed by clinical laboratory examination or imaging examination, age ≥18 years old, and all patients who signed informed consent. Exclusion criteria: serious complications such as gastrointestinal bleeding, gastric perforation, and pyloric obstruction, complicated with immune dysfunction or blood system disorder, complicated with hyperglycemia, hyperlipemia, and hypertension, complicated with malignant tumor or serious infection, mental disorder or mental illness, unable to cooperate with the scale survey, and pregnant and lactating women.

### 2.2. Intervention Methods

#### 2.2.1. The Control Group Received Traditional Nursing Measures. The Intervention Lasted for 2 Months

The main nursing measures were basic condition observation, to understand the characteristics of symptoms of chronic gastritis and gastric ulcer in patients, ward environmental nursing, routine admission health education, medication guidance, actively guide patients to maintain a reasonable schedule, inform patients of relevant matters needing attention during hospitalization, and give patients a health knowledge manual on chronic gastritis and gastric ulcer.

#### 2.2.2. The Study Group Received Standardized Nursing Intervention Combined with Mindfulness Stress Reduction Training. The Intervention Lasted for 2 Months

Standardized nursing intervention: according to the different conditions of patients, standardized nursing procedures were formulated, and the specific intervention measures were as follows. ① Before nursing: formed a standardized nursing intervention group, the group included the leading physician, the head nurse, and the responsible nurse, carried out special training for responsible nurses on chronic gastritis and gastric ulcer, clarified different division of labor, and carried out nursing intervention after the training was completed. ② Hospitalization period: (I) Medication guidance: nurses popularized the knowledge of chronic gastritis and gastric ulcer to patients, explained the causes, pathogenesis, specific treatment methods, prognosis, and other disease content, gave patients detailed guidance on the medication method, medication time, and dosage every time, informed patients of possible side effects of drugs, instructed patients to took drugs on time and in quantity, avoided sudden withdrawal of drugs, and avoided changing drugs without authorization. Medical staff explained to patients that once serious side effects of drugs occur, they should be informed immediately, and professional medical staff should change drugs or stop taking drugs. (II) Daily nursing: nurses made a detailed investigation on patients' eating habits and living conditions and made a detailed daily nursing plan. Patients should be given scientific and reasonable nutritional diet intervention. The foods in the diet should be rich in trace elements such as high protein and vitamins. The intake of acidic foods should be controlled. Oily, spicy, gas-producing, and irritating foods should be fasted. The purpose of eating on time and eating slowly should be strictly observed. The types of foods should be arranged reasonably to ensure the patients' balanced diet and adequate nutrition intake. Medical staff should supervise patients to develop healthy living habits in their daily life, arranged their work and rest time reasonably, ensure that patients have enough sleep, and remind patients to increase or decrease clothes appropriately according to temperature changes, so as to kept their stomach warm. (III) Sports nursing: nurses should reasonably arrange the way and time of exercise according to the individual situation of patients, encourage patients to go out and participate in group activities as much as possible, and guide patients to take reasonable aerobic exercise, such as nonstrenuous exercise such as walking after meals and Tai Chi, and accelerate blood circulation through aerobic exercise. (IV) Psychological nursing: nurses should increase the communication between nurses and patients, understand and meet the needs of patients as much as possible, know the sources of patients' negative emotions in detail, and instruct their families to pay more attention to the mental state of patients, so that patients could establish a healthy state of mind. At the same time, we could give patients psychological support and comfort through conversation, explain the harm of negative emotions, and adjust their psychological pressure, so that patients could maintain a good attitude towards life. ③ After discharge: followed up the patients until they fully recover. Urged patients to develop good living habits by telephone, instructed patients to check their stomach regularly, and informed patients of corresponding treatment methods in case of adverse reactions after discharge.

Mindfulness stress reduction training: according to the different conditions of patients, the mindfulness stress reduction training methods were formulated, nursing interventions for patients in a group manner, and the specific intervention measures were as follows. ① Week 1: explained the specific theory of mindfulness stress reduction training to patients, issued instruction manuals, organized 30-minute mindfulness breathing training teaching, guided patients to hold their breath, concentrated on breathing, kept regular breathing, listened to breathing sounds, and count the number of breaths, so that patients could gather their spirits to perceive the current environment and get rid of distractions. After training, explained patients' doubts and encouraged patients to communicate with each other. Twice a week. ② Week 2: instructed the patients to keep sitting posture, guided the patients to meditate, guided the patients to breathe with the rhythm of music, and perceived their own emotions. During meditation, patients need to bring mindfulness breathing and posture into meditation and observe thoughts and events emerging in their minds. Meditate for 40 min at a time. Twice a week. ③ Week 3: instructed the patient to meditate by the body scanning method, made the patient concentrate, started to scan the body consciousness from the foot, then transferred attention to all parts of the body slowly and systematically, scanned and meditated the body from bottom to top, and made the body relax completely. Every body scan was 30 min. Three times a week. ④ Week 4: while doing scanning meditation, nurses could also give Tai Chi guidance to patients. After meditation scanning, nurses could help the patient perform the first eight types of Tai Chi, explain the essentials of movement for patients, and guide them to exercise. The total time of meditation and Tai Chi exercise was 1 h, three times a week.

### 2.3. Observation Index

The general clinical data such as age, gender, course of disease, education level of the two groups were recorded.

Evaluation criteria of the curative effect. Cure: the clinical symptoms of chronic gastritis and gastric ulcer disappeared, and the original ulcer surface was completely healed by gastroscopy. Effective: the clinical symptoms of chronic gastritis and gastric ulcer basically disappeared, and the area of focus site in gastroscopy decreased by ≥50%. Ineffective: the clinical symptoms of chronic gastritis and gastric ulcer were not improved or even aggravated, and the area of focus site in gastroscopy decreased by <50% or not decreased. Total effective rate = (cure + effective)/total cases × 100%.

Self-rating anxiety scale (SAS) and self-rating depression scale (SDS) were used to evaluate patients' negative emotions. SAS and SDS have a total of 20 items and adopt a four-level scoring method, in which “1” has no or little time, “2” has a small part of time, “3” has quite a lot of time, and “4” has most or all time. Standard score = total rough score × 1.25. SAS score <50 indicates no anxiety, 50–59 was mild anxiety, 60–69 was moderate anxiety, and >69 was severe anxiety. SDS score <53 indicates no depression, 53–62 was mild depression, 63–72 was moderate depression, and >73 was severe depression. High scores of SAS and SDS indicate more negative emotions.

General self-efficacy scale (GSES) was used to evaluate patients' self-efficacy. There were 10 items in the scale, with a 4-level scoring method of 1–4 points, with a total score of 10–40 points, 10–20 points for low efficiency, 21–30 points for medium efficiency, and 31–40 points for high efficiency. High score of GSES means high self-efficacy.

Generic quality of life inventory-74 (GQOL-74) was used to evaluate patients' quality of life. There were 74 items in the questionnaire, including four dimensions of physical function, mental function, social function, and life state. There are 5 factors for physical function, mental function, social function, and 4 factors for life state. The total score of each dimension of the scale was 100 points. High score of GQOL-74 means a good quality of life.

The satisfaction questionnaire made by our hospital was used to evaluate the nursing satisfaction of patients, including the nurse's working ability, working attitude, help provided, and daily guidance. The total score was 100 points, and the survey results are divided into dissatisfied: <60 points, satisfied: 60–80 points, and very satisfied: >80 points, with total satisfaction rate = (very satisfied + satisfied)/total cases × 100%. The content validity index of the self-made satisfaction questionnaire was 0.90, and the internal consensus reliability coefficient of Cronbach's *α* was 0.91.

### 2.4. Statistical Analysis

SPSS 22.0 statistical software was used for processing, the counting data were expressed in (%), and the *χ*^2^ test was used for comparison. Measurement data are expressed in ($\bar{x}$ ± *s*), and comparison was made by the *t*-test. *P* < 0.05 was statistically significant.

## 3. Results

### 3.1. The General Data between the Two Groups

There were no significant differences in age, gender, course of disease, and education level of the two groups (*P* > 0.05), as given in Table 1.

### 3.2. The Nursing Efficiency between the Two Groups

The nursing effective rate of the study group (91.78%) was higher than the control group (79.45%) (*P* < 0.05), as given in Table 2.

### 3.3. The Negative Emotions between the Two Groups

After intervention, the SAS score and SDS score of the study group were lower than the control group (*P* < 0.05), as shown in Figure 1.

### 3.4. The Self-Efficacy between the Two Groups

After intervention, the GSES score of the study group was higher than the control group (*P* < 0.05), as shown in Figure 2.

### 3.5. The Quality of Life between the Two Groups

After intervention, the GQOL-74 scores of the study group were higher than the control group (*P* < 0.05), as shown in Figure 3.

### 3.6. The Nursing Satisfaction between the Two Groups

The nursing satisfaction rate of the study group (89.04%) was higher than the control group (75.34%) (*P* < 0.05), as given in Table 3.

## 4. Discussion

Chronic gastritis and gastric ulcer are common diseases of the digestive system, especially in today's fast-paced life and work. Due to living habits, diet, and environmental factors, the incidence of gastric ulcer and chronic gastritis is gradually increasing [9]. Although chronic gastritis and gastric ulcer generally do not bring life-threatening to patients, chronic gastritis and gastric ulcer often have different degrees of discomfort and a variety of bad emotions. As the disease progresses, the psychological status of patients deteriorates, which often seriously affects the quality of life of patients [10]. In the clinical treatment of chronic gastritis and gastric ulcer, gastric mucosal protection drugs are often used, which completely eradicate *Helicobacter pylori* and combine with proton pump inhibitors to maintain the gastric pH value. However, it is difficult to control the recurrence of the disease only by drug treatment. Therefore, in the treatment of chronic gastritis and gastric ulcer, not only should we pay attention to the scientific and rational use of drugs but also carry out scientific nursing intervention and find effective nursing intervention means to improve patients' living standards.

The results of this study showed that after standardized nursing intervention combined with mindfulness stress reduction training, patients with chronic gastritis and gastric ulcer have a good curative effect, less negative emotion, and higher self-efficacy. In our opinion, the possible reason is that standardized nursing can promote the further healing of gastritis and gastric ulcer and reduce the corresponding pain through medication guidance, daily nursing, sports nursing, psychological nursing, and follow-up after discharge, which is scientific and comprehensive, can effectively improve the comfort of patients and meet the health needs of patients to the greatest extent [11]. In the process of standardized nursing intervention, nurses explain the related knowledge of chronic gastritis and gastric ulcer in detail to help patients understand the symptoms, treatment procedures, precautions, and other information, so that patients can have a comprehensive understanding of their own diseases. Nurses guide and inform patients of possible side effects after medication, which is conducive to the return of digestive tract function to normal. Scientific daily nursing and exercise nursing can help patients develop good living habits; healthy and nutritious diet management can reduce the gastric mucosa from being damaged again and reduce the risk of disease recurrence. At the same time, aerobic exercise can accelerate blood circulation, contribute to gastrointestinal peristalsis and metabolism, and enhance the function of the digestive system. After the patient is discharged from hospital, the medical staff can prevent the patient from having gastric mucosal damage again by monitoring the patient to develop a healthy life schedule, which plays a positive role in promoting the complete recovery of the patient's disease [12]. Mindfulness stress reduction training can make patients accept themselves uncritically, face diseases correctly with a peaceful attitude, reduce the interference of bad thoughts, enhance the level of mindfulness, which can gradually enhance patients' physical adjustment ability and self-disease management ability, and lead patients to have the concept of self-regulation of diseases, thus having a good therapeutic effect [13]. In addition, for patients with chronic gastritis and gastric ulcer, because of the long course of disease, it is difficult to cure, and patients generally have anxiety and depression. With the aggravation and deterioration of the disease, the negative emotions of patients are also increasing, and the self-efficacy is also decreasing [14]. Self-efficacy refers to the degree of confidence that people can use their skills to achieve and complete a certain behavior goal, which can have an impact on people's physical and mental health [15]. Traditional treatment only focuses on gastrointestinal diseases, often ignoring the psychological state of patients, and the nursing effect has certain limitations. Therefore, it is necessary for nurses to stimulate patients' positive psychology in the process of nursing, so as to improve patients' confidence in recovery. Standardized nursing focuses on observing patients' psychological conditions and psychological counseling, which can give full play to patients' inherent potential, improve patients' behavior, cultivate patients' courage to face diseases, and improve patients' self-efficacy. At the same time, patients are given psychological support through conversation, and the harm of negative emotions is explained to them, so that patients can establish a happy state of mind and reduce psychological pressure [16]. Mindfulness stress reduction training can help patients with chronic gastritis and gastric ulcer to deal with their negative emotions correctly by guiding them to meditate and listen to breathing sounds. In addition, nurses guide patients to slowly and systematically shift their attention to various parts of the body and scan and meditate on the body from bottom to top, so that patients' body and mind are completely relaxed, reducing negative emotions and enhancing patients' self-efficacy [17].

For patients with chronic gastritis and gastric ulcer, most of them are given simple traditional nursing in the clinic, which can make patients know the disease knowledge and improve the clinical symptoms to a certain extent. However, the traditional nursing activities are single and one-sided, lacking systematic and comprehensive clinical services, and the nursing intervention effect was not good. The results of this study can reveal that standardized nursing intervention combined with mindfulness stress reduction training can improve patients' quality of life and nursing satisfaction. Standardized nursing intervention first formulates standardized nursing procedures according to patients' different needs and cognition and then takes targeted and effective nursing measures according to patients' eating habits, lifestyle, and psychological state. Standardized nursing can help patients understand the importance of taking drugs on time, give them scientific and reasonable nutrition recipes, reasonably arrange patients' exercise mode and time, relieve patients' psychological pressure and other nursing measures, so as to improve patients' self-control ability, help patients develop healthy living habits, help patients control digestive tract symptoms more effectively, and exert the best nursing effect as much as possible, promote patients' recovery, and improve their quality of life. Mindfulness stress reduction training mainly includes mindfulness breathing, experience exchange, meditation, music relaxation, and body scanning. This method can help patients with chronic gastritis, and gastric ulcer eliminates negative cognition of negative events, thus relieving the perceived pressure of patients and improving their physical and mental conditions. In the implementation of mindfulness stress reduction training, nursing staff can guide patients to concentrate on the present, awaken patients' inner focus on themselves, encourage patients not to suppress their inner thoughts, actively face the occurrence of diseases, eliminate distractions, relax their bodies and minds, and perceive diseases with an indifferent state of mind, which can have a positive impact on the improvement of living standards and nursing satisfaction [18]. It is worth mentioning that although mindfulness stress reduction training is developing rapidly in our country, the course quality, duration, and content of the program need to be improved, and the record of hard indicators needs to be improved. Therefore, we should summarize the clinical application experience at home and abroad, so as to further optimize the intervention measures of mindfulness stress reduction training.

## 5. Conclusion

Standardized nursing intervention combined with mindfulness stress reduction training has a good curative effect in patients with chronic gastritis and gastric ulcer, which is beneficial to reduce negative emotions, increase self-efficacy, improve quality of life, and improve nursing satisfaction.

## Figures and Tables

**Figure 1:** The negative emotions between the two groups. *Note*. Compared with before intervention, ^*∗*^*P* < 0.05; compared with the control group, ^#^*P* < 0.05.

**Figure 2:** The self-efficacy between the two groups. *Note*. Compared with before intervention, ^*∗*^*P* < 0.05; compared with the control group, ^#^*P* < 0.05.

**Figure 3:** The quality of life between the two groups. *Note*. Compared with before intervention, ^*∗*^*P* < 0.05; compared with the control group, ^#^*P* < 0.05.

**Table 1:** The general data between the two groups (%).

Group	Age (years)	Gender		Course of disease (years)	Education level		
		Male	Female		Primary school	Junior high school	High school or above
Control group (*n* = 73)	41.39 ± 7.32	44 (60.27%)	29 (39.73%)	2.57 ± 1.01	7 (9.59%)	30 (41.10%)	36 (49.32%)
Study group (*n* = 73)	40.81 ± 7.57	41 (56.16%)	32 (43.84%)	2.52 ± 1.16	8 (10.96%)	33 (45.21%)	32 (43.84%)
*t*/*χ*^2^ value	0.470	0.253	0.278	0.445			
*P* value	0.638	0.615	0.781	0.801			

**Table 2:** The nursing efficiency between the two groups (%).

Group	Cure	Effective	Ineffective	Total effective rate
Control group (*n* = 73)	31 (42.46%)	27 (3.99%)	15 (20.55%)	58 (79.45%)
Study group (*n* = 73)	43 (58.90%)	24 (32.88%)	6 (8.22%)	67 (91.78%)
*χ* ^2^ value				4.505
*P* value				0.034

**Table 3:** The nursing satisfaction between the two groups (%).

Group	Very satisfied	Satisfied	Dissatisfied	Total satisfaction rate
Control group (*n* = 73)	29 (39.73%)	26 (35.61%)	18 (24.66%)	55 (75.34%)
Study group (*n* = 73)	40 (54.79%)	25 (34.25%)	8 (10.96%)	65 (89.04%)
*χ* ^2^ value				4.679
*P* value				0.031

## Data Availability

The data used and/or analyzed during the current study are available from the corresponding author.
